The article "A randomized, double‐blind, controlled study evaluating the effects of two facial serums on skin aging" was retracted in 2026. Reasons: compromised peer review; original data or images not available; lack of ethics approval or compliance.

# A randomized, double‐blind, controlled study evaluating the effects of two facial serums on skin aging

**DOI:** 10.1111/srt.13522

**Published:** 2023-11-23

**Authors:** Daniel Banov, Maria Carvalho, Steve Schwartz, Robert Frumento

**Affiliations:** ^1^ Research and Development (R&D) Professional Compounding Centers of America (PCCA) Houston Texas USA; ^2^ International Research Services Inc. (IRSI) New York USA

**Keywords:** delivery/vectorization/penetration, formulation/stability, liposomal blend, skin aging, skin barrier, visual analog scale

## Abstract

**Background:**

Skin aging is a natural process that occurs because of oxidative stress. Facial skin aging is often concerning for individuals due to the exposure of the face.

**Objectives:**

To assess and compare the effects of two anti‐aging facial serums on the following characteristics associated with facial skin aging: fine lines/wrinkles, age spots, firmness, elasticity, texture, radiance, tone, lifting, clarity, and complexion.

**Methods:**

A 24‐week, double‐blind controlled study was conducted on 130 participants who were randomized into two groups: facial serum with Liposomal Blend and facial serum without Liposomal Blend. Clinical evaluations (Visual Analog Scale) and instrumental evaluations (Cutometer, SIAscope, and Clarity Pro image analysis) were performed at weeks 0 (baseline), 2, 4, 8, 12, and 24 to assess for changes in skin aging characteristics.

**Results:**

A total of 123 participants completed the study; participants that used the facial serum with Liposomal Blend had significantly greater improvements in skin aging characteristics compared to those that used the facial serum without Liposomal Blend. This study shows that Liposomal Blend is a vehicle with the ability to enhance the anti‐aging properties of the ingredients within the facial serum by facilitating its delivery into the underlying layers of the skin. Higher concentration of ingredients at the site of action could potentially lead to greater damage repair and improvements in signs of facial skin aging.

**Conclusion:**

By using Liposomal Blend, practitioners and pharmacists could potentially improve the delivery of the ingredients within their formulations into the skin, which may lead to increased treatment efficacy.

## 1 INTRODUCTION

Skin aging is a complex process that occurs naturally as a consequence of oxidative stress caused by Reactive Oxygen Species (ROS), a by‐product of cellular metabolism. The accumulation of ROS within cells can damage Deoxyribonucleic Acid (DNA) and proteins, which can halt proliferation and result in cell death.^1^ ROS also have the ability to upregulate the expression of pro‐inflammatory cytokines such as Interleukins (IL)−1, IL‐6, and Tumor Necrosis Factor‐alpha (TNF‐α), which can increase the activity of Matrix Metalloproteinases (MMPs), enzymes that degrade extracellular matrix within the dermis.^2^ Extracellular matrix provides structural support to the skin and is composed of collagen, a protein that contributes mass and tensile strength, and elastin, a protein with elastic characteristics.^1^ The decline in cell count and increased extracellular matrix degradation therefore causes alterations in the structure and function of the skin layers, resulting in skin aging.^2^

The article "A randomized, double‐blind, controlled study evaluating the effects of two facial serums on skin aging" was retracted in 2026. Reasons: compromised peer review; original data or images not available; lack of ethics approval or compliance.

The process of skin aging has an effect on the whole body. However, facial skin aging is often more concerning for individuals as the face is a part of the body that is visible to others.^3^ Characteristics associated with facial skin aging include: fine lines/wrinkles; alterations in skin firmness, elasticity, texture, and lifting; development of age spots; and alternations in skin tone, clarity, radiance, and complexion. Fine lines and wrinkles are folds in the skin caused by cell death and loss of extracellular matrix that provide support and structure to the skin.^4^ Skin firmness refers to the ability of the skin to resist change,^5^ while elasticity relates to the ability of the skin to return to its original shape upon deformation.^2^ Reduced skin firmness and elasticity are commonly observed in aging individuals as a result of the reduction in collagen and elastin content within their skin.^2^, ^5^ Texture, which refers to the degree of roughness on the skin surface, is affected by organization of the collagen fibers. A change in skin texture occurs with age because of collagen fibers reorganization, causing an increase in skin roughness.^6^ Lifting is a characteristic affected by thinning of the skin layers and loss of subcutaneous fat in regions below the dermis, resulting in sagging of the skin.^1^ Age spots are dark regions on the skin commonly found in sun‐exposed areas such as the face. As the skin ages, cell death hinders the body's ability to remove the pigments melanin and lipofuscin, resulting in pigments accumulation and the formation of age spots.^7^ The presence of these dark regions on the skin can affect an individual's skin tone and clarity. Tone is determined based on the pigmentation pattern of the skin,^8^ while clarity refers to the presence/absence of skin markings such as blemishes.^9^ Those with even tone and clear skin will have even distribution of pigments throughout the face, with no markings. Radiance is a term used to describe the level of skin brightness, while complexion is a general term that describes the overall appearance of the skin. An individual's complexion depends on a combination of factors such as skin texture, tone, radiance, and clarity.^9^

The article "A randomized, double‐blind, controlled study evaluating the effects of two facial serums on skin aging" was retracted in 2026. Reasons: compromised peer review; original data or images not available; lack of ethics approval or compliance.

Though genetics play a major role in facial skin aging, environmental factors such as ultraviolet radiation from sunlight exposure, smoking, stress, poor diet, and alcohol can accelerate the aging process and worsen facial skin aging characteristics.^10^ When these characteristics become too prominent, individuals often search for cosmetic interventions in an attempt to diminish signs of skin aging.^3^ The objective of this study is to assess and compare the effects of two anti‐aging facial serums, one with Liposomal Blend, and one without Liposomal Blend, on the following characteristics associated with facial skin aging: fine lines/wrinkles, age spots, firmness, elasticity, texture, radiance, tone, lifting, clarity, and complexion. Liposomal Blend is a permeation enhancer that is used topically as a vehicle in cosmetics and pharmaceutical formulations. It consists of proprietary liposomal components designed to enhance the delivery of substances into the underlying layers of the skin. It includes 0.05% to 5% of one or more phospholipids; 1% to 20% of Pracaxi oil that is used as a permeation enhancer in the natural composition and that decreases irritation and provides hydration and restores a cutaneous permeability of skin; 0.1% to 3% of one or more skin lipids; 1% to 10% of a butter having linoleic acid and linolenic acid; and 10% to 90% of purified water, wherein a substantial portion of liposomes of the natural liposomal composition are about 5 to 20 microns.^11^ The liposomal constituents have potentials to attach to skin surfaces and fuse with the lipid bilayer, facilitating delivery of ingredients into the skin.^12^, ^13^

The two facial serums were developed for the purposes of preventing and improving the appearance of aging skin, and contain the following ingredients with proposed anti‐aging activities: caffeine, pracaxi oil, *Plukenetia volubilis* seed oil, *Carthamus tinctorius* seed oil, palmitoyl tripeptide‐5, hexapeptide‐9, acetyl‐dipeptide‐1 cetyl ester, niacinamide, and methylsulfonylmethane (MSM). Caffeine is a naturally occurring substance with antioxidant activity. When applied to human skin fibroblasts, cells that produce collagen, caffeine helps to reduce ROS‐mediated cellular damage and necrosis.^14^ Pracaxi oil, extracted from the seeds of *Pentaclethra macroloba* tree found in the Amazon forest, contains large amounts of fatty acids that play an essential role in the construction of cell membranes within the stratum corneum and epidermis. The fatty acids from pracaxi oil also have anti‐inflammatory properties and could potentially protect the skin from damage by ultraviolet radiation.^15^ *Plukenetia volubilis* seed oil, extracted from a shrub plant native to the Amazon as well, contains omega‐3 and omega‐6 fatty acids with antioxidant activity. Studies have shown that *Plukenetia volubilis* extract also has the ability to facilitate fibroblast migration.^16^ *Carthamus tinctorius* (safflower) seed oil contains fatty acids with antioxidant and anti‐inflammatory activities.^17^ Palmitoyl tripeptide‐5 is a peptide that exerts its anti‐aging effects by activating Tissue Growth Factor (TGB)‐β, which increases collagen synthesis within the skin.^18^, ^19^ Hexapeptide‐9 has the ability to facilitate skin regeneration^10^ while acetyl‐dipeptide‐1 cetyl ester was used for its skin soothing effects.^20^ Niacinamide (vitamin B3) is a water soluble vitamin that is a precursor to coenzymes involved in many metabolic reactions within the skin. Results from studies conducted with topical niacinamide show that in addition to having antioxidant activities, this vitamin can help improve skin texture, as well as the appearance of wrinkles and age spots.^21^, ^22^ MSM is a compound that contributes sulfur to replenish glutathione levels within the body, resulting in a reduction in ROS‐mediated cellular damage as glutathione is a free radical scavenger.^23^

The article "A randomized, double‐blind, controlled study evaluating the effects of two facial serums on skin aging" was retracted in 2026. Reasons: compromised peer review; original data or images not available; lack of ethics approval or compliance.

## 2 MATERIALS AND METHODS

A 24 weeks, randomized, double‐blind controlled study was conducted to assess and compare the effects of two anti‐aging facial serums, one serum with Liposomal Blend, and another serum without Liposomal Blend, on characteristics associated with facial skin aging. This study was conducted in Port Chester, NY by International Research Services Inc., and informed consent was obtained from all study participants.

### 2.1 Study design

A total of 130 female participants were enrolled in this study based on the inclusion and exclusion criteria displayed in Table 1. Enrollment was followed by a washout period of 1 week in which participants were instructed to wash their face with Camay soap and warm water, at least two times a day, and to apply Purpose lotion SPF 15 daily. The use of any topical facial treatment products was prohibited during the washout period and throughout the course of this study.^24^ Aside from the Camay soap and Purpose lotion SPF 15, participants were allowed to continue the use of color cosmetics provided that their packaging did not make any claims regarding moisturizing and/or anti‐aging. At the end of the washout period, participants were randomized into two groups: facial serum with Liposomal Blend (group A) and facial serum without Liposomal Blend (group B), with 65 participants in each group. At the baseline visit, participants were provided the assigned facial serum and were shown how to apply the product to the entire face, including the areas under the eye. Participants were instructed to apply the serum twice daily for a period of 24 weeks. In order to record compliance, participants were given a diary to record the times that they used the product for every day of the study. It was established that participants would be disqualified if compliance was lower than 80%.

The article "A randomized, double‐blind, controlled study evaluating the effects of two facial serums on skin aging" was retracted in 2026. Reasons: compromised peer review; original data or images not available; lack of ethics approval or compliance.

**TABLE 1:** Inclusion and exclusion criteria for enrollment of the study participants.

Inclusion criteria	Exclusion criteria
Healthy females between 39 to 65 years of age at the time of enrollment. Able to understand and willing to complete a brief personal history, review and sign an informed consent document, and follow all study instructions. Lines/wrinkles in the periorbital area with a score greater than 2 cm and less than 8 cm on a standard 10 cm visual analog scale (VAS). Willing to come to the observation site without makeup. Willing to continue use of all regular brands of color cosmetics provided they do not make any moisturizing or anti‐aging claims. Willing to refrain from using new facial products other than the assigned test materials.	Pregnant, breast‐feeding, or planning a pregnancy during the course of the study. Initiated the use of topical or oral prescription steroids and/or anti‐inflammatory medications within 30 days of study enrollment. Participating in any other clinical studies. Known allergies to personal care product(s) (self‐reported). History of sensitivity to skin treatment products. Any dermatologic disorders that may interfere with evaluation of test product performance. Any condition(s) apparent at entry or recognized after entry that are likely to invalidate a subject's consent to participate in this study and/or limit the ability of a subject to regularly attend all study visits or to comply with all other protocol requirements such as: diseases, injuries, alcoholism, drug abuse, psychosis, antagonistic personality, poor motivation, infirmity disability, other problems that may be emotional, intellectual, psychological or social. An employee of the testing facility or other testing firms/laboratories, cosmetic or raw goods manufacturers or suppliers.

Visits to the testing facility occurred at week 0 (baseline), 2, 4, 8, and 12 for all participants, while a subgroup of participants were evaluated through to week 24. Participants were instructed to wash their face at least 1 to 2 h prior to each visit. Upon arrival, participants remained at room temperature for at least 15 min to allow the skin to equilibrate to ambient indoor conditions prior to evaluation.^24^ Clinical and instrumental evaluations were then performed to measure for changes in skin aging characteristics, from baseline, following the use of the assigned facial serum. A self‐assessment questionnaire was also conducted at baseline and each subsequent visit to assess the participant's perception of product use. The questionnaire, as displayed in Table 2, consists of 10 statements to which participants were instructed to answer based on whether or not they agreed with the specific statement.

The article "A randomized, double‐blind, controlled study evaluating the effects of two facial serums on skin aging" was retracted in 2026. Reasons: compromised peer review; original data or images not available; lack of ethics approval or compliance.

**TABLE 2:** Self‐assessment questionnaire.

Statements
Product use reduced the facial skin discoloration (age spots)
Product use reduced the appearance of periorbital fine lines/wrinkles
Product use reduced the appearance of perioral fine lines/wrinkles
Product use improved facial skin firmness
Product use improved facial skin elasticity
Product use improved facial skin texture/smoothness
Product use increased facial skin radiance
Product use improved facial skin tone
Product use improved facial complexion health
Product use improved facial skin clarity

### 2.2 Clinical evaluations

The facial skin of all participants was clinically graded by a trained evaluator using the Visual Analog Scale (VAS), a tool that can be utilized to quantify subjective characteristics,^25^ such as those shown in Figure 1. VAS scales have been widely used in previous studies to examine the effects of various anti‐aging formulations on facial skin aging.^24^, ^26^ Evaluators were instructed to specify their level of agreement to a statement by indicating a position along a 10 cm line between the two end‐points, one end being 0 and the other end being 10. Signs of photo‐aging can be categorized as follows: mild (1 to 3.9), moderate (4 to 6.9), or severe (7‐10).^24^ The same evaluator performed all assessments throughout the study.

**FIGURE 1:** Visual Analog Scales (VAS) for skin aging clinical evaluations.

### 2.3 Cutometer

The Cutometer MPA580 (Courage and Khazaka Electronic GmbH; Köln, Germany) is an instrument that allows the characterization of the mechanical properties of the skin such as firmness and elasticity.^27^, ^28^ This instrument consists of a pressure generator connected to a hand‐held probe with a 4 mm opening. Once the probe establishes contact with the skin surface, a constant negative pressure from the generator stretches and pulls the skin into the opening of the probe. After a specified time interval of suction, the probe then releases the skin and allows it to recover in shape.^27^ This suction and release procedure, which is typically repeated for at least 3 cycles, was performed on one side of the face, in the region of the cheek, at baseline and each subsequent visit. The investigators used an individual face map to identify the same facial area for measurements at each visit. Changes in skin shape that occur during the suction and release cycles are detected and recorded every 0.1 s.^29^ by an optical system within the probe, which consists of an infrared light source transmitting to a receptor.^27^ The intensity of the light transmitted is dependent on the amount of skin that penetrates the probe during suction and release, creating a strain‐time curve that depicts the degree of skin deformation in millimeters (mm) over time. The curve is then used in waveform analysis by the Cutometer software to measure the amount of skin raised by the suction probe (i.e., height of the curve); the amount of force required to induce the stretch; and the rate at which the skin returns to equilibrium, generating the waveform variables R0 and R5,^28^ which represent skin firmness and elasticity, respectively.

The article "A randomized, double‐blind, controlled study evaluating the effects of two facial serums on skin aging" was retracted in 2026. Reasons: compromised peer review; original data or images not available; lack of ethics approval or compliance.

### 2.4 SIAscope

The skin content of melanin and collagen was quantified via spectrophotometric intracutaneous analysis using the Cosmetrics SIAscope (Astron Clinica Ltd.; Cambridgeshire, United Kingdom), an instrument that consists of a probe connected to a laptop computer. The probe is hand‐held and is first placed in direct contact with the skin surface on one side of the face. The light‐emitting diodes inside of the probe then shine a spectrum of visible and infrared light onto the skin at discreet wavelengths of 400 to 1000 nm.^24^, ^30^ The light establishes contact with the skin surface and is absorbed by chromophores such as melanin^31^ scattered by molecules such as collagen^32^ or reflected. The probe is programmed to capture the reflected light and information is relayed to the SIAscope software on the laptop computer.^30^ The software performs a series of calculations to generate a high resolution image that shows the melanin and collagen in the skin at each wavelength, along with chromophore maps that were retrieved up to 2 mm in depth and 11 mm in circumference. These chromophore maps were used to determine the concentration and distribution of melanin and collagen within the skin layers.^31^ Previous studies have shown that the method of chromophore mapping can be used to assist in the diagnosis of malignant skin conditions such as melanoma,^30^, ^31^ as well as to assess for changes in characteristics associated with skin aging.^24^, ^33^ Chromophore mapping using the Cosmetrics SIAscope was performed on all participants in this study at baseline, weeks 8, 12, and 24. As before, the investigators used an individual face map to identify the same facial area for measurements at each visit.

The article "A randomized, double‐blind, controlled study evaluating the effects of two facial serums on skin aging" was retracted in 2026. Reasons: compromised peer review; original data or images not available; lack of ethics approval or compliance.

### 2.5 Clarity Pro

The Clarity Pro (BrighTex Bio‐Photonics; San Jose, CA) is an instrument with the ability to capture and generate a three‐dimensional (3D) image of the face using multi‐spectral lighting.^34^ The facial skin of 20 participants from each group was analyzed using the Clarity Pro imaging system at baseline, weeks 4, 8, 12, and 24. Participants were instructed to position their chin on the instrument's chin rest, with the forehead touching a stopper to ensure that there was a constant and reproducible distance between the camera and each participant's face. Frontal and lateral (45°) white and blue light images of the face were then captured by three cameras with specialized lenses that operate in conjunction with one another.^35^ These images were further analyzed by a computer software within the instrument using mathematical algorithms that allow for quantification of skin aging characteristics, as well as visualization of the skin's condition on and beneath the facial skin surface.^34^, ^35^ The Clarity Pro has been used in previous studies also as an objective method for measuring facial skin redness associated with rosacea, ^35^ and wrinkle characteristics associated with skin aging.^34^

## 3 RESULTS

A total of 123 female participants completed the study, with 63 participants in group A and 60 participants in group B. Of the seven participants that discontinued the study, two participants experienced mild facial itching and redness, while the remainder participants withdrew for personal reasons unrelated to product use. According to the daily diary, compliance was over 90% for all the 123 participants. Demographics information of the study participants is shown on Table 3. The majority of the participants were purposely Caucasian as facial skin aging is more prominent in this race group. African Americans, Hispanics and multi‐ethnic participants were also included in this study though the results obtained were grouped and analyzed altogether. Although it would have been interesting to include men in this study to observe the permeation enhancer in relationship to skin thickness, the primary goal of this study was to compare the effects of two anti‐aging facial serums in female subjects, who commonly suffer changes in skin aging characteristics due to hormonal imbalances, particularly around menopause. Mean ± standard deviation (SD) of clinical and instrumental scores were calculated for each group at baseline and at each visit. Differences in scores between baseline and subsequent time points were calculated for both groups. Scores obtained from clinical evaluations and instrumental analyses were compared between groups using an un‐paired t‐test, with *p* ≤ 0.05 denoting statistical significance. Chi‐squared analysis was performed to compare scores obtained from the self‐assessment questionnaire.

The article "A randomized, double‐blind, controlled study evaluating the effects of two facial serums on skin aging" was retracted in 2026. Reasons: compromised peer review; original data or images not available; lack of ethics approval or compliance.

**TABLE 3:** Demographics information of the study participants.

Characteristics	Group A (Mean ± SD)		Group B (Mean ± SD)		*p‐*value
Height (inches)	63.57 ± 2.79		63.42 ± 2.74		0.771
Weight (pounds)	166.00 ± 42.65		165.45 ± 37.79		0.940
Age (years)	57.61 ± 6.88		56.70 ± 6.83		0.459
Race	*n* (%)		*n* (%)		0.139
	Caucasian	45 (71.4%)	Caucasian	46 (75.4%)	
	African American	15 (23.8%)	African American	7 (11.5%)	
	Hispanic	3 (4.8%)	Hispanic	7 (11.5%)	
	Multi‐Ethnic	0 (0.0%)	Multi‐Ethnic	1 (1.6%)	

### 3.1 Clinical evaluations

VAS was used to quantify change in skin aging characteristics. An increase in mean VAS scores from baseline was observed at weeks 2 and 4 visits for the majority of characteristics examined. Differences between the two groups were not statistically significant (*p* > 0.05) for all characteristics, with the exception of skin clarity, where mean difference in VAS scores from baseline was significantly lower for group B (−0.01 ± 0.72) in comparison to group A (0.26 ± 0.73), *p* = 0.042 (Figure 2). At the week 8 visit, group A had a reduction in mean VAS scores for all characteristics, while fluctuations in scores were observed for group B. Furthermore, group A's score for skin texture was significantly lower than group B at weeks 8 (*p* = 0.021) and 12 (*p* = 0.037) visits, as displayed in Figure 3. Difference in skin texture scores between the two groups continued to be significant at week 24 (*p* = 0.012), along with group A having significantly lower scores than group B in terms of radiance (*p* = 0.004), tone (*p* = 0.017), lifting (*p* = 0.014), clarity (*p* = 0.047), and complexion health (*p* = 0.020).

**FIGURE 2:** Clinical evaluations for skin clarity: VAS mean scores for Groups A and B at weeks 2 to 24, in comparison to baseline.

**FIGURE 3:** Clinical evaluations for skin texture/smoothness: VAS mean scores for Groups A and B at weeks 2 to 24, in comparison to baseline.

### 3.2 Cutometer

When comparing skin firmness, a reduction in mean scores from baseline was observed for both groups at each visit following the start of treatment. Mean difference in scores from baseline for group A (−0.21 ± 0.07) was significantly lower than group B (−0.16 ± 0.06) at week 24, *p* = 0.022. When comparing skin elasticity, mean scores for group A increased from baseline at each subsequent visit, while group B scores increased at weeks 2, 4, and 8, with no change at week 12, and a reduction in score at week 24. Significant differences were detected between the groups at week 24, with participants in group A (0.14 ± 0.35) having higher scores than those in group B (−0.07 ± 0.28), *p* = 0.044, as displayed in Figure 4.

The article "A randomized, double‐blind, controlled study evaluating the effects of two facial serums on skin aging" was retracted in 2026. Reasons: compromised peer review; original data or images not available; lack of ethics approval or compliance.

**FIGURE 4:** Cutometer analysis for elasticity in the skin: mean scores for Groups A and B at weeks 2 to 24, in comparison to baseline.

### 3.3 SIAscope

The SIAscope was used to quantify melanin and collagen levels in the skin. Results show an initial reduction from baseline in melanin levels for groups A (−7.96 ± 16.61) and B (−9.76 ± 15.77) at week 8, with no significant differences between the two groups, *p* = 0.537. Melanin levels continued to decrease for group A (−8.87 ± 16.21) at week 12, while a slight increase in level was detected for group B (−8.32 ± 18.82), *p* = 0.879. Though both groups had an increase in melanin at week 24, group A levels (5.55 ± 11.97) were significantly higher than group B (−7.70 ± 13.84), *p* = 0.003. Collagen levels within the skin also fluctuated between weeks 8 and 12 for both groups. However, as the study progressed, the collagen levels detected within the skin of participants in group A (2.78 ± 11.17) were significantly higher than that of group B (−6.25 ± 11.11) at week 24, *p* = 0.017, as displayed in Figure 5.

**FIGURE 5:** SIAscope analysis for collagen in the skin: mean scores for Groups A and B at weeks 8 to 24 in comparison to baseline.

### 3.4 Clarity Pro

Selected results from Clarity Pro image analysis are shown on Table 4. Difference in mean scores between baseline and subsequent visits were calculated for groups A and B. Based on the images captured, following the use of the facial serum with Liposomal Blend for 24 weeks, the participants had a 54.46% reduction in total number of wrinkles, 22.94%, 23.07%, and 38.34% reduction in wrinkle width, length, and severity, respectively.

**TABLE 4:** Clarity Pro analysis for total wrinkles, average wrinkle length and width, and fine lines: Mean scores for Groups A and B at weeks 4 to 24, in comparison to baseline (*p*‐value).

	Total lines/wrinkles		Average wrinkle length		Average wrinkle width		Fine lines	
Characteristics	Group A	Group B	Group A	Group B	Group A	Group B	Group A	Group B
Week 4	‐0.79	‐4.27	0.31	‐0.9	0.13	0.07	3.21	‐2.45
Week 8	‐6.42	‐11.9	‐3.78	‐0.98	‐0.08	0.12	‐5.53	‐10.3
Week 12	‐14.88	‐26.42	‐1.48	‐7.76	0.14	‐0.75 (0.003)	‐9.31	‐15.89
Week 24	‐35.11	‐2.8	‐20.76	0.06 (0.001)	‐1.44	‐0.43 (0.030)	‐27.17	6.56 (0.047)

### 3.5 Self‐assessment questionnaire

The perception of the study participants with regards to the facial serums improved as a function of time (product use) for both groups, as displayed in Table 5. The majority of participants (> 50%) agreed that both facial serums improved facial skin firmness and texture/smoothness at every visit through week 24.

The article "A randomized, double‐blind, controlled study evaluating the effects of two facial serums on skin aging" was retracted in 2026. Reasons: compromised peer review; original data or images not available; lack of ethics approval or compliance.

**TABLE 5:** Percentage of affirmative responses with regards to product use (self‐assessment questionnaire).

	Week 2			Week 4			Week 8			Week 12			Week 24		
Statements	Group A	Group B	*p*‐value	Group A	Group B	*p*‐value	Group A	Group B	*p*‐value	Group A	Group B	*p*‐value	Group A	Group B	*p*‐value
Product use reduced the facial skin discoloration (age spots)	22.20%	13.30%	**0.045**	29.00%	24.60%	0.315	36.50%	27.90%	0.303	41.00%	37.30%	0.186	29.40%	43.50%	0.384
Product use reduced the appearance of peri‐orbital fine lines/wrinkles	47.60%	38.30%	0.31	53.20%	45.60%	0.222	57.10%	47.50%	0.461	63.90%	57.60%	0.676	58.80%	69.60%	0.429
Product use reduced the appearance of peri‐oral fine lines/wrinkles	34.90%	25.00%	0.169	43.50%	36.80%	0.529	44.40%	36.10%	0.407	50.80%	40.70%	0.303	52.90%	52.20%	0.25
Product use improved facial skin firmness	65.10%	53.30%	0.224	72.60%	50.90%	**0.005**	69.80%	62.80%	0.348	75.40%	57.60%	**0.051**	82.40%	73.90%	0.739
Product use improved facial skin elasticity	41.30%	36.70%	0.197	54.80%	42.10%	0.258	52.40%	52.50%	0.185	57.40%	50.80%	0.273	70.60%	65.20%	0.756
Product use improved facial skin texture/smoothness	74.60%	71.70%	0.607	74.20%	66.70%	0.536	81.00%	78.70%	0.734	82.00%	76.30%	0.387	94.10%	78.30%	0.069
Product use increased facial skin radiance	42.90%	41.70%	0.826	43.50%	50.90%	0.646	61.90%	52.90%	0.475	65.60%	49.20%	0.123	52.90%	60.90%	0.305
Product use improved facial skin tone	44.40%	36.70%	0.074	50.00%	43.90%	0.466	52.40%	49.20%	0.485	65.60%	55.90%	0.376	35.30%	56.50%	0.122
Product use improved facial complexion health	49.20%	60.00%	0.309	48.40%	56.10%	0.591	63.50%	63.90%	0.354	67.20%	61.00%	0.349	70.60%	65.20%	0.692
Product use improved facial skin clarity	47.60%	38.30%	0.334	47.50%	40.40%	0.668	52.40%	49.20%	0.845	62.30%	47.50%	0.146	29.40%	56.50%	0.11

Bold *p*‐values denote statistically significant results.

## 4 DISCUSSION

Alterations in skin aging characteristics following the use of the two facial serums were assessed using VAS (clinical evaluations); Cutometer, SIAscope, and Clarity Pro image analysis (instrumental evaluations).

### 4.1 Clinical evaluations

An increase in mean VAS is indicative of skin aging. Results of this study show worsening of almost all examined skin characteristics at weeks 2 and 4 for both groups as mean VAS scores were higher in comparison to baseline. Skin clarity (Figure 2) was the only characteristic by week 4 that showed a significant difference between the participants that used the facial serum with Liposomal Blend (group A) and without Liposomal Blend (group B). Skin texture/smoothness, on the other hand, showed significant results from week 8 towards the end of the study, with clear improvements by group A in comparison to group B, as shown in Figure 3. By week 24, the participants that used the facial serum with Liposomal Blend showed significant improvements of the following skin characteristics: texture/smoothness, radiance/luminosity, skin tone, lifting, complexion health, and clarity. The only skin characteristics that did not show statistically significant results by the clinical evaluations were wrinkles, age spots, and elasticity/firmness. These characteristics were reassessed by instrumental analysis, as discussed below.

The article "A randomized, double‐blind, controlled study evaluating the effects of two facial serums on skin aging" was retracted in 2026. Reasons: compromised peer review; original data or images not available; lack of ethics approval or compliance.

### 4.2 Cutometer

Skin firmness and elasticity scores were calculated based on analysis of the waveforms generated following skin suction with the cutometer.^28^ Lower scores are indicative of improved skin firmness, while higher scores are indicative of improved skin elasticity. The lower skin firmness score and higher skin elasticity scores observed for group A at week 24 show that the skin of participants that used the facial serum with Liposomal Blend was more firm and elastic in comparison to those that used the facial serum without Liposomal Blend.

### 4.3 SIAscope

The SIAscope was used to quantify melanin and collagen content within the skin. Melanin is a pigment that determines the color of an individual's skin. The fluctuations in melanin levels for groups A and B throughout the course of the study could potentially be due to variations in participants’ exposure to sunlight as this is an external factor that can influence melanin levels in the skin.^36^ Collagen is a fibrous protein that provides support and strength to the skin. Reduced collagen synthesis can lead to dermal atrophy and is characteristic of aging skin.^37^ The higher collagen levels detected for group A at week 24 could potentially lead to enhanced skin firmness and elasticity for participants using the facial serum with Liposomal Blend.

### 4.4 Clarity Pro

Images captured with the Clarity Pro were used to assess for change in total lines/wrinkles, characteristics associated with the lines/wrinkles, age spots, radiance, and complexion health. Results from Clarity image analysis showed statistically significant mean difference in complexion health scores between groups A and B at week 8, with improvements in skin complexion detected for participants in group B, *p* = 0.03. Differences between the two groups were also seen for average wrinkle width (*p* = 0.003) and complexion health (*p* < 0.001) at week 12, in which group B was superior to group A. However, improvement in scores for group B were not maintained for the remainder of the study and, at week 24, group A's scores for average wrinkle length (*p* = 0.001), average wrinkle width (*p* = 0.030), and fine lines (*p* = 0.047) were superior to that of group B. These results show that by the end of the study, participants that used the facial serum with Liposomal Blend had significant reduction in fine lines, as well as the length and width of the lines/wrinkles compared to those that used the facial serum without Liposomal Blend.

The article "A randomized, double‐blind, controlled study evaluating the effects of two facial serums on skin aging" was retracted in 2026. Reasons: compromised peer review; original data or images not available; lack of ethics approval or compliance.

## 5 CONCLUSION

The primary goal of anti‐aging formulations is to prevent and reduce, as much as possible, the visible signs of facial skin aging.^3^ Though these skin aging characteristics may appear on the surface of the face, damage to the skin is often deeper, involving the epidermal layers below the stratum corneum as well as the dermis.^10^ Adequate penetration of ingredients from anti‐aging formulations into the underlying layers of the skin is therefore necessary to improve characteristics associated with skin aging. Though the two facial serums examined in this study contain identical ingredients, participants that used the facial serum with Liposomal Blend had significantly greater improvements in skin aging characteristics compared to those that used the facial serum without Liposomal Blend. Results from this study show that Liposomal Blend is a vehicle with the ability to enhance the anti‐aging properties of the ingredients within the facial serum by facilitating its delivery into the underlying layers of the skin. Higher concentration of ingredients at the site of action could potentially lead to greater prevention and improvements in signs of facial skin aging. By using Liposomal Blend, practitioners and pharmacists could potentially improve the delivery of the ingredients within their formulations into the skin, which may lead to increased treatment efficacy.

## FINANCIAL DISCLOSURE

The authors Daniel Banov and Maria Carvalho are affiliated with Professional Compounding Centers of America (PCCA), the manufacturer of the Liposomal Blend. Daniel Banov is a full‐time employee at PCCA and Maria Carvalho is a consultant for PCCA. The authors Steve Schwartz and Robert Frumento are affiliated with International Research Services Inc. (IRSI) and have no commercial or financial relationship with PCCA. IRSI received financial compensation for the execution of this study.

## Data Availability

Data sharing is not applicable to this article as no new data were created or analyzed in this study.
